The article "Directional Dependence of Experimental Trunk Stiffness: Role of Muscle-Stiffness Variation of Nonneural Origin" was published in 2020. Journal: Appl Bionics Biomech.

# Directional Dependence of Experimental Trunk Stiffness: Role of Muscle-Stiffness Variation of Nonneural Origin

**DOI:** 10.1155/2020/8837147

**Published:** 2020-12-09

**Authors:** Sadok Mehrez, Hichem Smaoui

**Affiliations:** ^1^Department of Mechanical Engineering, College of Engineering at Al Kharj, Prince Sattam bin Abdulaziz University, 11942, Saudi Arabia; ^2^LASMAP, Tunisia Polytechnic School, University of Carthage, Tunisia; ^3^Department of Civil and Environmental Engineering, Faculty of Engineering, King Abdulaziz University, Jeddah, Saudi Arabia; ^4^LAMOED, Ecole Nationale d'Ingénieurs de Tunis, University of Tunis El Manar, Tunisia

## Abstract

Trunk stiffness is an important parameter for trunk stability analysis and needs to be evaluated accurately. Discrepancies regarding the dependence of trunk stiffness on the direction of movement in the sagittal plane suggest inherent sources of error that require explanation. In contrast to the common assumption that the muscle stiffness remains constant prior to the induction of a reflex during position perturbations, it is postulated that muscle-stiffness changes of nonneural origin occur and alter the experimental trunk stiffness, causing it to depend on the sagittal direction. This is confirmed through reinterpretation of existing test data for a healthy subject, numerical simulation, and sensitivity analysis using a biomechanical model. The trunk stiffness is determined through a static approach (in forward and backward directions) and compared with the model stiffness for assumed scenarios involving deactivated muscles. The difference in stiffness between the opposite directions reaches 17.5% without a preload and decreases when a moderate vertical preload is applied. The increased muscle activation induced by preloads or electrical stimuli explains the apparent discrepancies observed in previous studies. The experimental stiffness invariably remains between low and high model-stiffness estimates based on extreme scenarios of the postulated losses of muscle activation, thereby confirming our hypothesis.

## 1. Introduction

The trunk stiffness is an important parameter used in studying trunk postural control and stability [1–4]. Spinal instability, which is a frequent cause of lower back pain and other health disorders, highlights the need for accurate evaluation of human trunk stiffness [5–7]. The determination of translational or (equivalently) rotational trunk stiffness has been the subject of several experiments involving sudden position perturbations [2, 8, 9]. The measured trunk stiffness depends on various factors. Some are controllable physical factors related to the design of the experiment, such as the subject posture, perturbation duration, and perturbation direction. Others are associated with the data interpretation and processing and depend on the adopted hypotheses and the models used to calculate the experimental stiffness [9–13]. In addition to experiments, numerical models of the trunk have been developed for the analysis and simulation of the trunk behavior [3, 14, 15]. Models that capture the details of this behavior may be useful for the interpretation and explanation of test results [8, 16]. The present work addresses the dependence of the trunk stiffness on the perturbation direction, which has been investigated experimentally [4, 5, 7] and was recently found to be significant [5, 7]. However, different protocols [4, 5] lead to contrasting assessments of this directional dependence in the sagittal plane. Moreover, no elaborate explanation has been provided for the disagreements. The objective of the present study was to investigate the sagittal-plane dependence of the trunk stiffness using numerical modeling and experimental data [17].

The sagittal directional dependence of the trunk stiffness, which was demonstrated in [5], was not evident in previous investigations. In [4], where stiffness was measured along various directional angles for standing subjects exerting voluntary horizontal preloads, the difference between the forward and the backward sagittal stiffness was negligible (2%). Subsequent studies on the sagittal-plane stiffness [3, 17, 18] tended to ignore the directional dependence. The stiffness relative to the forward and backward perturbations was assumed to be identical, and the data were treated without distinction between the directions of perturbation. Multidirectional tests involving sitting subjects [5] revealed differences of up to 15% between the forward and the rearward stiffness. The difference decreased when the subjects were exposed to an electrical stimulus [7] that tended to increase muscle activation. This suggests that augmented muscle activation resulting from external stimuli, e.g., an electric excitation [7], a horizontal preload [3, 4, 18], or a vertical preload [17], is a factor that should be considered in the investigation of the directional dependence. The tests reported in [17], which were originally intended for investigating the trunk stability, involved a subject lifting loads. The test results included information on the effects of the carried loads on the trunk stiffness and its directional dependence. However, these effects were not visible because the data were treated without distinction between the directions of perturbation. The directional dependence can be analyzed using the same data, by separately treating the forward and rearward perturbation results.

The measured trunk stiffness is a combination of varying components that must be dissociated to obtain a rigorous interpretation of test data. The transient stiffness is generally determined during short transient trunk position perturbations [5, 7, 18], which involves passive, intrinsic [3, 19], and paraspinal reflex stiffness [20]. The intrinsic and reflexive components can be separated using displacement-controlled actuation, ending the perturbation before the reflexive reaction begins [3, 21]. The intrinsic part is commonly calculated by solving a dynamic identification problem [20, 22], where the stiffness effect is coupled with inertial and damping forces. The stiffness effect can be further separated from the dynamic effects using the static approach [17] based on two states: the pre- and postperturbation states. An end-state stiffness (ESS) of the trunk, composed of the passive and the intrinsic stiffness only, is deduced from the two motionless states immediately preceding and following position perturbations, which are both free of reflex activation [17]. This yields a net stiffness that depends on measurements performed at the initial and final states only. Furthermore, in both the static and dynamic approaches [5, 7, 22], the intrinsic stiffness was considered to be invariant during the position perturbation, under the assumption that the muscle active forces remain constant. Consequently, the forward stiffness and the rearward stiffness were considered to be identical. The argument underlying the assumption of muscle-force invariance is that trunk-position perturbations in flexural tests are designed to occur entirely before the induction of neural activation and presumably before any change in muscle activation [17]. However, the assumption of force invariance is not supported by experimental evidence [3, 22, 23]. Conceptually, the intrinsic trunk stiffness in the sagittal plane is posture-specific. At a given posture, it is a resultant of skeletal and muscle-tendon stiffness relative to that posture and should be indifferent to posterior events affecting the trunk, such as changes in the position, regardless of direction. The muscle stiffness is directly dependent on the forces governed by muscle recruitment at the given posture. Under static conditions, the active muscle stiffness is considered to be proportional to the active force [24–26]. With such an unequivocal characterization of the muscle stiffness, the trunk stiffness should mechanically be independent of the direction despite the anatomic asymmetry in the sagittal plane. However, the issue of trunk-stiffness variability arises in connection with measurement. Force and position measurements must be performed at the reference posture and one or more perturbed postures where the muscle stiffness may differ.

During position perturbation, even before the induction of a paraspinal reflex, an activated muscle may undergo a stiffness reduction due to excessive shortening or a high shortening velocity [24, 27, 28]. The hypothesis posed in this paper is that muscle-stiffness losses of nonneural origin affect the experimental trunk stiffness and result in its sagittal direction dependence. A numerical model that accounts for changes in the muscle stiffness and allows calculation of the trunk ESS separately in the forward and backward directions was used in the present investigation, together with available trunk test data [17]. Because of the trunk anatomical asymmetry in the sagittal plane, the stiffness changes differed between forward and rearward perturbations.

## 2. Materials and Methods

### 2.1. Trunk Test

The trunk experiment, which provided the data used in the present study, was performed in the Kevin P. Granata Biomechanics Laboratory at Virginia Tech and described in [17]. It determines the ESS, for forward and backward position perturbations, of one healthy male subject standing upright with pelvic motion blocked. The experiment was originally designed to study the effects of vertical preloads on the static stability of the spine. A rotary servomotor shaft was pin-attached eccentrically to a rod connected by a ball-and-socket joint (at the T10 level) to a harness fixed on the subject's chest. The horizontal forces developed at the joint, and the induced displacements were recorded during a sequence of ±1.5 mm displacements. The forces were measured using an in-line force transducer with a resolution of 0.725 N/mV. The displacements were determined according to rotational angles measured using an optical encoder attached to the servomotor shaft. The signals for the forces and the displacements were sampled at 1000 Hz and processed with a low-pass filter. A series of tests was performed with the subject supporting his own weight only or carrying additional weights of 133.5, 267, and 400 N. To minimize unwanted oscillations, the subject is instructed to stiffen his neck, and the weights are symmetrically suspended from his shoulders by long ropes.

The subject held an emergency safety button to shut down the servomotor at any time during the test. The experimental trunk ESS was calculated using the force data recorded for the anterior and posterior position perturbations.

### 2.2. Numerical Model

The biomechanical model (Figure 1) determines the static response of the trunk to external loads. It is a static, multibody type model comprising the spine, the rib cage, and 174 muscles [14, 29]. The vertebrae, intervertebral discs, sternum, and ribs are represented by beam elements, and the ligaments are modeled as linear springs. The skeletal geometry is reconstructed according to the stereographic method described in [30], on the basis of X-ray images of the subject standing in an upright posture. The independent variables are the muscle active forces and the nodal displacements, which constitute the basic model output. The muscle force-length relationship [24, 31] defines the maximum physiological active force *F*_UB_ as a function of the muscle length *L* and maximum active force at rest *F*_0max_. The minimum active force *F*_LB_, i.e., the tonus, and maximum force *F*_0max_ of a muscle are constants that are proportional to its largest physiological cross-sectional area (Equations (1) and (2)) and are given as follows [14]:

(1) $$\begin{array}{c} F_{0\max}=c\text{PCSA}, \end{array}$$

(2) $$\begin{array}{c} F_{\text{LB}}=\alpha F_{0\max}. \end{array}$$

Here, the input model parameters are defined as follows: PCSA—the largest physiological cross-sectional area of the muscle, *c*—a constant given in [17], and *α*—the muscle tonus ratio deduced from experimental data [17].

In the model, each muscle is represented by its active force *F* and force-dependent active stiffness *k*_*a*_, which is determined as follows:

(3) $$\begin{array}{c} k_{a}=q\frac{\text{F }}{L}, \end{array}$$

where *q* is a constant dimensionless input parameter [19] and *L* represents the muscle length, which depends on the displacements.

The muscle length is determined from the calculated positions of the muscle insertion points. The displacements are subject to physiological kinematic constraints [32] restricting intervertebral motion.

The trunk-response calculation involves two sets of independent variables: the nodal displacements and the muscle active forces. The muscle recruitment problem is formulated as a constrained minimization problem (Equation (4)) and solved using the MATLAB function *fmincon*. It involves finding the muscle forces that minimize the Euclidean norm of the muscle stress vector while maintaining equilibrium with the applied loads and satisfying the physiological kinematic constraints [32] and any prescribed displacements.

The muscles active forces and the trunk displacements, which are the model outputs, are repeatedly updated by solving an equilibrium problem (Equation (5)) integrated within the recruitment problem (Equation (4)):

(4) $$\begin{array}{c} \begin{array}{cc} \underset{\left\{F\right\}}{\mathrm{minimize}\;} & \left\|\sigma \left(\left\{F\right\}\right)\right\|,\\ \text{subject to} & F_{\text{LB}}^{m}\leq F_{m}\leq F_{\text{UB}}^{m}\left(L_{m}\left(\left\{U\left(\left\{P^{k}\right\},\left\{F\right\}\right)\right\}\right)\right),\;1\leq m\leq N. \end{array} \end{array}$$

Here, the symbols are defined as follows: *N* is the number of modeled muscles, {*F*} is the vector of muscle forces, *m* is the muscle reference index, *F*_*m*_ is the force of the *m*^th^ muscle, *σ* is the vector of muscle stresses, {*P*^*k*^} is the vector of applied loads at the *k*^th^ load increment, *U* is the displacement vector, *L*_*m*_ is the length of the *m*^th^ muscle, *F*_LB_^*m*^ is the muscle minimal active force (tonus), and *F*_UB_^*m*^ is the muscle maximal active force.

The equilibrium problem (Equation (5)) consists of minimizing the total mechanical potential energy of the trunk system subject to the external loads, the muscle forces, and the kinematic constraints:

(5) $$\begin{array}{c} \begin{array}{cc} \min & \left(\frac{1}{2}{\left\{\Delta U^{k}\right\}}^{T}\left[K^{k}\right]\left\{\Delta U^{k}\right\}-{\left\{P^{k}\right\}}^{T}\left\{\Delta U^{k}\right\}\right),\\ \text{subject to} & U_{\text{LB},ij}\leq \left(U_{i}^{k}+\Delta U_{i}^{k}\right)-\left({\text{U}}_{j}^{k}+\Delta U_{j}^{k}\right)\leq U_{\text{UB},ij}\;1\leq i<j\leq \text{NDV}. \end{array} \end{array}$$

Here, the symbols are defined as follows: *k* is the loading increment index; {*P*^*k*^} is the vector of applied forces; {*U*^*k*^} is the displacement vector at the *k*^th^ increment; *U*_*i*_^*k*^ and *U*_*j*_^*k*^ are the displacement components of two adjacent vertebrae; NDV is the number of degrees of freedom associated with the vertebrae; [*K*^*k*^] is the system stiffness matrix, which depends on {*U*^*k*^} and {*F*}; Δ*U*_*i*_^*k*^ and Δ*U*_*j*_^*k*^ are the displacement increments relative to preceding equilibrium position; and *U*_LB,*ij*_ and *U*_UB,*ij*_ are the lower and upper bounds on relative displacement [32] between two adjacent vertebrae.

This quadratic programming problem is solved using the MATLAB *quadprog* function.

### 2.3. Muscle-Tendon Behavior

The experimental trunk ESS introduced in Section 2.1 is governed by the state of muscle-tendon complexes during the perturbation. Because the trunk settles in the postperturbation state, the effective trunk stiffness should be defined according to the forces and displacements in this state.

To determine the forward and the backward trunk stiffness separately, the unilateral behavior of the muscle-tendon complex is taken into consideration. Clearly, the tendon cannot withstand compression. It is stretched while carrying tensile forces; in their absence, it is relaxed, and the active force in the corresponding muscle vanishes. Additionally, the tension vanishes when the maximum shortening velocity is exceeded, even for active muscles [24]. The tension reductions due to muscle-tendon length variations cause losses in the muscle active stiffness even though the neural activation remains constant. These changes in muscle stiffness should be considered in the numerical model.

In the following, the “state” of the tendon or muscle refers to whether it is stretched or unstretched and whether it is subjected to tension or is force-free. The stretching is defined relative to a generic reference length that depends on the activation and contraction dynamics. It is common [24] to consider the length at rest *L*_0_ as the reference. In this study, the reference length is defined as the preperturbation length, on an approximate basis.

At the outset of perturbation, the body is in a natural state where muscles are all activated and in a state of tension. The muscles are activated at least at the tonus level. After perturbation, there are three possible muscle-tendon states. In the first state, the muscle remains stretched and fully maintains its active force and stiffness. In the second, the muscle remains stretched, but the active force decreases because of the high shortening velocity. In the third state, the tendon is relaxed owing to shortening; thus, the muscle loses its stiffness, and the force in it vanishes.

### 2.4. Model Stiffness Calculation

The trunk stiffness of the model is determined as the ratio of a horizontal force increment to the calculated induced displacement. For a given preperturbation trunk state, the calculation involves two steps. First, the recruitment problem is solved for the muscle activations consistent with the given trunk state. Second, a specified horizontal force increment is added to the forces of Step 1. Then, the equilibrium problem is solved using the muscle stiffness derived from the preperturbation activations obtained in Step 1, while treating the T10 displacement as free. To approach the test conditions, the force increment is set to a value that induces a 3 mm displacement. For a more realistic estimation, the muscle-stiffness values should be those recorded immediately after perturbation (preceding the induction of the reflex), because the trunk settles in the static postperturbation state. In this end state, the muscle active forces and elongations remain at their eventual unknown postperturbation levels, which determine the trunk reaction to be used in the model trunk stiffness calculation.

An approximate assessment of the end state of the trunk muscles is performed first by running the recruitment problem subject to the preperturbation conditions. The muscle-tendons that are shortened during the displacement perturbation are identified and are considered as potentially inactive. Depending on the investigative purpose, some of these candidates are retained as inactive, with the others being treated as active at their preperturbation levels. In the subsequent equilibrium problem, the inactive muscles are considered to withstand no forces and to no longer develop stiffness. The equilibrium problem is solved subject to the force increment while considering only the retained active muscles, followed by a straightforward calculation of the trunk stiffness.

By adopting appropriate criteria for defining the postperturbation status of muscles, lower and upper estimates of the trunk stiffness can be obtained. For instance, assuming scenario 1 for all muscle-tendons preserves the muscle stiffness, leading to an upper estimate. Alternatively, an overprediction of tendon relaxation contributes to underestimating the trunk stiffness. An extreme scenario is one where all shortening muscles are deactivated. Interestingly, the idea of selective muscle deactivation provides a quantitative indicator of the influence of an individual muscle or muscle group, which is obtained by calculating its contribution to the trunk stiffness.

### 2.5. Model Parameters

The muscles' insertion points are determined according to the graphic localization specified in [14, 32]. The adopted muscle PCSA values are taken from average anthropometric data reported in [14]. With regard to muscle behavior, two parameters remain to be estimated. The first is the constant *q* which is widely reported in the literature [33, 34]. It is determined through model calibration [17] and found to be equal to 10. Regarding the second, i.e., the tonus, conclusive relevant information is lacking, and it is unclear to what extent the tonus level is muscle-specific. The tonus levels are estimated according to tonus values determined through model calibration. Additionally, a sensitivity analysis is performed for the trunk stiffness as a function of tonus. Using the chosen tonus levels, numerical upper and lower estimates of the forward and backward experimental trunk stiffness values*K*_*f*,exp_ and *K*_*b*,exp_ are obtained. The upper estimates correspond to the maximum trunk stiffness values *K*_*f*,max_ and *K*_*b*,max_, determined with all the muscle-tendons remaining activated during perturbation. The lower estimates correspond to the reduced trunk stiffness values *K*_*f*,min_ and *K*_*b*,min_, determined while excluding from the calculation the muscle-tendons undergoing shortening during perturbation. Because the upper estimates *K*_*f*,max_ and *K*_*b*,max_ are calculated according to the same set of active muscles, they are identical. They are both denoted as *K*_max_ (*K*_max_ = *K*_*f*,max_ = *K*_*b*,max_).

If the true set of activated muscles for a given direction of movement were known and used in the model, the resulting (realistic) trunk stiffness estimate would necessarily lie between the maximum and minimum ones. These two extreme estimates are said to form a bracketing of the realistic estimate. Moreover, the trunk stiffness calculated according to a realistic set of deactivated muscles should be a closer approximation of the experimental stiffness. Thus, the latter is expected to be bracketed by the minimum and maximum model estimates, provided that the model is sufficiently accurate. This bracketing of the experimental stiffness can serve as an indicator of the quality of the numerical model. It is used here to assess the choice of muscle tonus levels treated as control parameters. Therefore, it is relevant to analyze the sensitivity of the trunk stiffness results to these parameters.

For a meaningful assessment of the tonus influence, the muscles are divided according to the PCSA and length, into three classes assumed to share a common ratio of the tonus to the maximum active force. Hence, muscles having a PCSA larger than 120 mm^2^ are assigned to class C3. The muscles with a PCSA of 120 mm^2^ or less and length greater than 200 mm are classified as C2, and the remaining muscles belong to class C1. The retained model tonus is a combination of three tonus ratios (associated with the three classes), verifying that the intervals ([*K*_*f*,min_, *K*_*f*,max_]) and ([*K*_*b*,min_, *K*_*b*,max_]) are larger than the 99% confidence interval for the experimental stiffness (Table 1).

## 3. Results

### 3.1. Experimental Results

The trunk stiffness was evaluated for forward and backward position perturbations using the experimental data. For each trunk experiment, 10 position perturbations are retained for calculating the trunk stiffness. The averages, standard deviations, and 99% confidence intervals for the experimental trunk stiffness in the forward and backward directions are presented in Table 1.

### 3.2. Model Results

The muscle-tendons that are shortened during position perturbations are presented in Table 2 together with the relative contribution of each muscle group to the trunk stiffness, averaged over the selected series of lifted loads. The observed changes in the muscle force distribution patterns associated with the variations in the series of loads are relatively small. This justifies focusing on the averages instead of dealing with load-specific results.

Groups 1 and 2 shorten exclusively in flexion. The shortening for group 1 (2) lies between 1.12 and 1.16 mm (0.37 and 1.08 mm, respectively). Many groups are found to shorten during extension only, and others undergo shortening during movement in either direction. The cumulative contribution of groups 1 and 2 represents 37% of *K*_*f*,max_. The muscles omitted in Table 2 remain activated and contribute 62.1% of the forward stiffness.

Muscles that shorten exclusively during backward perturbation belong to the *erector spinae*, with most shortenings between 0.7 and 0.9 mm. Their contribution to the rearward stiffness amounts to 39%. Furthermore, the *multifidus* alone accounts for 6.3% of the trunk stiffness, with most shortenings between 0.31 and 0.94 mm. Muscle groups 3–5, which undergo shortening in both anterior and posterior perturbations, together contribute less than 1% in either direction. The remaining muscles, which are omitted from Table 2, are kept active, and their contribution to the backward stiffness is 53.45%.

### 3.3. Analysis of Results

For the subject carrying no load, the experimental trunk stiffness is 17.5% larger in the forward than in the backward direction. As the load is increased, the difference between the rearward and the forward stiffness decreases and reaches zero at a carried load of approximately 200 N. Beyond this load, the rearward stiffness becomes larger than the forward stiffness.

The trunk experiment was designed such that the perturbation occurs while neural activations remain unchanged. Because the perturbation is preceded by a sustained state of equilibrium, all muscles are active prior to perturbation. Thus, during muscle-tendon shortening, the tendon condition may belong to either scenario 1 or 3. Model results indicate that most preperturbation muscle forces are less than 50 N for all loading levels. The elongations due to a 50 N force remain under 0.5 mm for most tendons [35–37]. This suggests that millimeter-scale shortenings occurring during the trunk test represent significant shortening magnitudes. Thus, relaxation leading to a loss of stiffness in some muscles during perturbation is not excluded.

The lists of deactivated muscles (Table 2) based on the adopted elongation criterion appear meaningful. For instance, groups 1 and 2—the main muscles responsible for spinal flexion—are shortened exclusively during forward perturbation. Through their sustained passive flexion during the test, they are expected to shorten while undergoing concentric contraction. Their important flexural role is illustrated by their cumulative contribution exceeding 1/3 of the trunk maximal stiffness. The muscle groups 3–5 contribute very little to the trunk flexion as their function is not associated with the spine flexion. The *psoas major*, which is usually recruited for thigh and hip flexion, makes the largest contribution, possibly because it interferes with spine flexion despite the subject's hip attachment. Likewise, the *quadratus lumborum* is recruited for extension, lateral flexion, and thoracic rotation. Both groups are clearly dissociated from flexural behavior. The muscle contributions should be considered as approximate sensitivity indicators. The cumulative contributions are calculated as sums of individual contributions, ignoring the interactions that may lead to an overestimation of the actual contribution of multiple groups acting simultaneously.

Muscles that shorten exclusively during posterior perturbation belong to groups 6–10, which are responsible for extension. They contribute over a third of the rearward trunk stiffness. They are naturally expected to shorten while undergoing concentric contraction. The *multifidus* muscles help maintain spine stability but are also recruited during extension. The muscle groups that shorten during both anterior and posterior perturbations together contribute only 1% of the extensional stiffness. Groups 3 and 5 are known for their secondary role in spinal extension, which explains their deactivation in backward perturbation. Their contribution is minimal but exceeds that of the *psoas major*, which plays no role in extension.

Table 3 presents the model-generated trunk stiffness lower and upper estimates based on assumed sets of inactive muscles, which provide a bracketing of the experimental trunk stiffness for the series of applied loads.

### 3.4. Sensitivity to Tonus Level

The tonus combination (15%, 28%, and 36%) labeled T1, which is associated with classes C1, C2, and C3, respectively, yields a narrow bracketing (Table 3) of the experimental stiffness. The sensitivity of the model trunk stiffness to the tonus is analyzed by varying the tonus ratio by ±4% in each class while keeping it constant for the other classes, resulting in six additional tonus combinations labeled T2–T7. For each combination, the minimum and the maximum trunk stiffness is recalculated for all the series of loads. For the *i*^th^ combination, i.e., Ti, the forward (backward) minimum stiffness is denoted as *K*_*f*,min,Ti_ (*K*_*b*,min,Ti_), and the maximum stiffness is denoted as *K*_max,Ti_. The sensitivity results are presented in Figures 2–4.

For all the tonus values, the experimental and the extremum model stiffness increases with the supported load, while the experimental stiffness is always between the extreme model values. The sensitivity of both the maximum and the minimum stiffness to the tonus almost vanishes for class C2 in both forward and backward perturbations. It also vanishes for the minimum backward stiffness for class C1. The sensitivity is low for the minimum forward and backward stiffness for class C3. For the remaining cases, i.e., the maximum stiffness for classes C1 and C3 and minimum forward stiffness for class C1, the model stiffness is significantly sensitive to the tonus. Among the explored tonus combinations, T4 provides the narrowest bracketing of the experimental forward trunk stiffness.

## 4. Discussion

As the trunk stiffness is a key parameter in the study of spine stability, accuracy and rigor in its evaluation are important. Discrepancies in trunk test data with regard to the dependence of the trunk stiffness on the direction in the sagittal plane [3–5, 17] raise questions regarding this dependence and the definition of experimental trunk stiffness. The dependence of the sagittal stiffness on the direction was found to be significant in [5] for subjects in a sitting posture. However, standing subjects who were tested during voluntary thoracic exertions exhibited nearly identical trunk stiffness in the forward and rearward directions [4]. The sagittal directional dependence was ignored in [3, 17, 21]. This followed from the argument that the muscle stiffness and consequently the trunk stiffness remained constant in the absence of a reflex reaction during a short perturbation, implying that the trunk stiffness was identical for opposite directions despite the anatomical asymmetry in the sagittal plane. In contrast, muscle-tendon behavior is known [24] to exhibit possible active stiffness changes of kinematic, nonneural origins. The major hypothesis posed in this paper is that these changes occur during test position perturbations in the absence of a reflex reaction and are responsible for the directional sagittal dependence of the measured trunk stiffness.

Support of this hypothesis involves numerous assumptions associated with the experimental protocol and the numerical model. A major assumption is that the sagittal trunk-stiffness dependence on the direction is not intrinsic but is associated with measurement. Ideally, the trunk stiffness is posture-specific and should be indifferent to position perturbations. In this sense, it would be independent of the perturbation direction despite the anatomical asymmetry. However, its experimental evaluation requires measurements at distinct time instants and postures where stiffness is likely to be different. It is common to assume the trunk stiffness to remain constant before the induction of the paraspinal reflex [3, 17, 21]. However, while muscle neural activations are kept constant before the reflex induction, which is defendable and can be verified from force measurements [17], the muscle active stiffness may vary owing to nonneural causes, such as the loosening of tendons or an excessive muscle shortening velocity. The main hypothesis of the present work is that these variations in stiffness, coupled with the anatomical asymmetry, are at the origin of the directional dependence. The loss in muscle stiffness was exclusively attributed to the loosening of the tendon. According to the simulation results, the average shortening velocity in all cases remained below 15% of the maximum shortening velocity. This suggests that velocity was not a determining factor of the muscle deactivation. A more rigorous tracking of muscle elongations and rates of shortening would require a dynamic model incorporating detailed muscle-tendon contraction dynamics. The deactivation criterion, considering that a muscle loses its activation if it merely undergoes shortening during the perturbation, does not accurately capture the complex muscle contraction behavior. However, it should be noted that this limitation was not detrimental to the accuracy of the stiffness calculations. It only affected the width of the bracketing interval.

The adopted static approach has the merit of isolating the stiffness component from the inertial and damping effects. It is based on the assumption that the pre- and postperturbation states are static for the trunk as a whole. The fact is that, while the attachment at T10 is at rest, the movement of the other parts of the trunk (the head and the suspended masses) is not restrained. Hence, preventive measures are taken to minimize undesirable movements. For this reason, long ropes are used to suspend the masses, and the subject is instructed to stiffen his neck to avoid unwanted head oscillations. The preperturbation state can justifiably be considered as wholly static because it is preceded by a phase involving no stimulus. The force signal is composed of the constant preperturbation static reaction in addition to the noise. As for the postperturbation state, its departure from a wholly static one is not excluded. Any persistent dynamic effect should be reflected in the reaction force at T10. The postperturbation force signal is composed of the static reaction superposed to the noise and any oscillatory reaction force. Before the induction of a paraspinal reflex, the latter component exclusively represents the reaction associated with the trunk dynamic effects, captured at T10. From inspection of the recorded T10 force signals, the variable part of the signal is found to be similar in pattern and magnitude to the preperturbation noise. In other words, the postperturbation dynamic effects are practically insignificant, which justifies the assumption of the static state. Further confirmation of the static assumption can be obtained through displacement measurement at nonrestrained locations using sensors or image processing [38–40].

The multiplicity of preload cases enlarges the set of relevant data used in the study. However, the data being specific to a single subject represents a limitation of the study at this stage. The participation of a statistically representative number of subjects in future experiments will provide for statistical relevance.

Examination of the influence of lifted loads on the difference between forward and rearward stiffness is pertinent for the comparison with previous work. The lifted loads are known to generally increase the activation levels in muscles [17, 41] like the horizontal preload in [4] and the electrical stimulus in [7]. In Vette et al. [5, 7], the difference dropped from 15% [5] to 11% due to low electrical stimulation [7]. Likewise, as shown in Table 1, it fell from 17.5% without a carried load to 4.9% and 0% for the subject supporting weights of 133.5 N and near 200 N, respectively. Thus, the insignificant difference reported in [4] can be explained by the effect of preloads which could reduce the difference to less than 2%.

## 5. Conclusions

In this study, in contrast with the common assumption of muscle-stiffness invariance, stiffness reductions of nonneural origin during the trunk test were demonstrated to affect trunk stiffness values significantly and to lie at the root of the directional dependence of the sagittal stiffness. The investigation is based on the retreatment of trunk test raw data (separately for forward and backward perturbations), combined with simulations performed using a numerical model specific to the same subject. The static technique is employed to separate the stiffness component from the dynamic effects. The results elucidate the apparent discrepancies in the reported differences [4, 5] between the forward and the backward stiffness through the role of increased muscle activation induced by a preload [3, 4, 18] or an electric stimulus [7].

## Figures and Tables

**Figure 1:** Trunk model comprising the spine, the thoracic cage, and 174 muscles.

**Figure 2:** Bracketing of (a) forward and (b) backward trunk stiffness with respect to the load for tonus levels T2 (11%, 28%, and 36%) and T3 (19%, 28%, and 36%) for classes C1, C2, and C3, respectively.

**Figure 3:** Bracketing of (a) forward and (b) backward trunk stiffness with respect to the load for tonus levels T4 (15%, 28%, and 32%) and T5 (15%, 28%, and 40%) for classes C1, C2, and C3, respectively.

**Figure 4:** Bracketing of (a) forward and (b) backward trunk stiffness with respect to the load for tonus levels T6 (15%, 24%, and 36%) and T7 (15%, 32%, and 36%) for classes C1, C2, and C3, respectively.

**Table 1:** Experimental stiffness results.

	*K*_*f*,exp_		99% CI	*K*_*b*,exp_		99% CI	Δ*K* (%)
Trunk loading (N)	*μ* (N/mm) (*p* < 0.001)	SD (N/mm)		*μ* (N/mm) (*p* < 0.001)	SD (N/mm)		
350	2.41	(0.11)	[2.32; 2.50]	2.05	(0.11)	[1.96; 2.14]	17.5
483.5	2.54	(0.11)	[2.45; 2.63]	2.42	(0.09)	[2.35; 2.49]	4.9
617	3.00	(0.13)	[2.90; 3.10]	3.13	(0.10)	[3.05; 3.21]	–4.1
750	3.19	(0.10)	[3.10; 3.27]	3.47	(0.13)	[3.36; 3.58]	–8

*μ*: mean value; SD: standard deviation; CI: confidence interval for the mean value; Δ*K*: 100(*K*_*f*,exp_ − *K*_*b*,exp_)/*K*_*b*,exp_.

**Table 2:** Muscles shortened following forward and backward position perturbations and their contribution to the trunk stiffness.

Muscle group		Forward perturbation		Backward perturbation	
#	Name	Muscle designation^∗^	%*K*_*f*,max_	Muscle designation^∗^	%*K*_*b*,max_
1	Rectus abdominis	RA	18.4		
2	External oblique	EO2; EO5; EO6	18.6		
3	Thoracic multifidus	tmf_L1; tmf_L2	0.1	tmf_L3; tmf_L4; tmf_L5	0.5
4	Psoas major	pL1VB; pL1TP; pL1-L2IVD; pL2TP; pL2-L3IVD; pL3TP; pL3-L4IVD; pL4TP; pL4-L5IVD	0.6	pL5TP; pL5VB	0.05
5	Quadratus lumborum	T12-I,3; T12,1-I,3; T12,2-I,3; T12,3-I,3; I,3-L1; I,3-L3; I,2-L4	0.2	T12,1-I,2; L2-12,1; L3-12,1; L3-12,2; L3-12,3; L4-12,3; I,2-L2; I,3-L2; I,1-L3; I,2-L3	0.4
6	Longissimus thoracis			LT3; LT4; LT5; LT6; LT7; T8; LT9; LT10; LT11; LT12	22.9
7	Iliocostalis lumborum pars thoracis			IT5; IT6; IT7; IT8; IT9; IT10; IT11; IT12	10.0
8	Longissimus thoracis pars lumborum			l1; l2; l3; l4; l5	2.6
9	Iliocostalis lumborum pars lumborum			I1; I2; I3; I4	3.8
10	Multifidus			m1s; m1t1; mlt2; mlt3; m2s; m2t1; m2t2; m2t3; m3s; m3t1; m3t2; m3t3; m4s; m4t1; m4t2; m4t3; m5s; m5t1; m5t2; m5t3	6.3

^∗^Abbreviations are taken from [14].

**Table 3:** Numerical bounds on the trunk stiffness in forward and backward perturbations.

Trunk loading (N)	*K*_max_ (N/mm)	*K*_*f*,min_ (N/mm)	*K*_*b*,min_ (N/mm)
350	3.14	1.90	1.37
483.5	3.43	2.10	1.43
617	3.75	2.31	1.49
750	4.06	2.54	1.55

## Data Availability

The data results are included in the manuscript.

## References

[1] Vazirian M., Shojaei I., Tromp R. L., Nussbaum M. A., Bazrgari B. (2016). Age-related differences in trunk intrinsic stiffness. *Journal of Biomechanics*.

[2] Hendershot B., Bazrgari B., Muslim K., Toosizadeh N., Nussbaum M. A., Madigan M. L. (2011). Disturbance and recovery of trunk stiffness and reflexive muscle responses following prolonged trunk flexion: influences of flexion angle and duration. *Clinical Biomechanics*.

[3] Moorhouse K. M., Granata K. P. (2007). Role of reflex dynamics in spinal stability: intrinsic muscle stiffness alone is insufficient for stability. *Journal of Biomechanics*.

[4] Gardner-Morse M. G., Stokes I. A. (2001). Trunk stiffness increases with steady-state effort. *Journal of Biomechanics*.

[5] Vette A. H., Masani K., Wu N., Popovic M. R. (2014). Multidirectional quantification of trunk stiffness and damping during unloaded natural sitting. *Medical Engineering & Physics*.

[6] Ruoxun F., Jie L., Jun L., Weijun W. (2019). Presentation of an approach on determination of the natural frequency of human lumbar spine using dynamic finite element analysis. *Applied Bionics and Biomechanics*.

[7] Vette A. H., Wu N., Masani K., Popovic M. R. (2015). Low-intensity functional electrical stimulation can increase multidirectional trunk stiffness in able-bodied individuals during sitting. *Medical Engineering & Physics*.

[8] Shahvarpour A., Shirazi-Adl A., Larivière C., Bazrgari B. (2015). Trunk active response and spinal forces in sudden forward loading–analysis of the role of perturbation load and pre-perturbation conditions by a kinematics-driven model. *Journal of Biomechanics*.

[9] Shojaei I., Suri C., van Dieën J. H., Bazrgari B. (2018). Alterations in trunk bending stiffness following changes in stability and equilibrium demands of a load holding task. *Journal of Biomechanics*.

[10] Shahvarpour A., Shirazi-Adl A., Larivière C., Bazrgari B. (2015). Computation of trunk stability in forward perturbations—effects of preload, perturbation load, initial flexion and abdominal preactivation. *Journal of Biomechanics*.

[11] Wong A. Y., Kawchuk G., Parent E., Prasad N. (2013). Within-and between-day reliability of spinal stiffness measurements obtained using a computer controlled mechanical indenter in individuals with and without low back pain. *Manual Therapy*.

[12] Wong A. Y., Parent E. C., Dhillon S. S., Prasad N., Kawchuk G. N. (2015). Do participants with low back pain who respond to spinal manipulative therapy differ biomechanically from nonresponders, untreated controls or asymptomatic controls?. *Spine*.

[13] Miller E. M., Bazrgari B., Nussbaum M. A., Madigan M. L. (2013). Effects of exercise-induced low back pain on intrinsic trunk stiffness and paraspinal muscle reflexes. *Journal of Biomechanics*.

[14] Christophy M., Senan N. A. F., Lotz J. C., O’Reilly O. M. (2012). A musculoskeletal model for the lumbar spine. *Biomechanics and Modeling in Mechanobiology*.

[15] Moalla F., Mehrez S., Najar F. Dynamic identification of human trunk behavior as a diagnosis tool for pathologic problems.

[16] Khoddam-Khorasani P., Arjmand N., Shirazi-Adl A. (2020). Effect of changes in the lumbar posture in lifting on trunk muscle and spinal loads: a combined in vivo, musculoskeletal, and finite element model study. *Journal of Biomechanics*.

[17] Mehrez S., Smaoui H., Ben Salah F. Z. (2012). A biomechanical model to simulate the effect of a high vertical loading on trunk flexural stiffness. *Computer Methods in Biomechanics and Biomedical Engineering*.

[18] Lee P. J., Rogers E. L., Granata K. P. (2006). Active trunk stiffness increases with co-contraction. *Journal of Electromyography and Kinesiology*.

[19] Bergmark A. (2009). Stability of the lumbar spine: a study in mechanical engineering. *Acta Orthopaedica Scandinavica*.

[20] Cholewicki J., Simons A. P., Radebold A. (2000). Effects of external trunk loads on lumbar spine stability. *Journal of Biomechanics*.

[21] Granata K. P., Slota G. P., Bennett B. C. (2004). Paraspinal muscle reflex dynamics. *Journal of Biomechanics*.

[22] Moorhouse K. M., Granata K. P. (2005). Trunk stiffness and dynamics during active extension exertions. *Journal of Biomechanics*.

[23] van den Hoorn W., Cholewicki J., Coppieters M. W., Klyne D. M., Hodges P. W. (2020). Trunk stiffness decreases and trunk damping increases with experimental low back pain. *Journal of Biomechanics*.

[24] Zajac F. E. (1989). Muscle and tendon: properties, models, scaling, and application to biomechanics and motor control. *Critical reviews in biomedical engineering*.

[25] Brown S. H., McGill S. M. (2005). Muscle force–stiffness characteristics influence joint stability: a spine example. *Clinical Biomechanics*.

[26] Colombini B., Nocella M., Bagni M. A., Griffiths P. J., Cecchi G. (2010). Is the cross-bridge stiffness proportional to tension during muscle fiber activation?. *Biophysical Journal*.

[27] Jones D. A. (2010). Changes in the force–velocity relationship of fatigued muscle: implications for power production and possible causes. *The Journal of Physiology*.

[28] Zivkovic M. Z., Djuric S., Cuk I., Suzovic D., Jaric S. (2017). Muscle force-velocity relationships observed in four different functional tests. *Journal of Human Kinetics*.

[29] Stokes I. A. F., Gardner-Morse M. (1995). Lumbar spine maximum efforts and muscle recruitment patterns predicted by a model with multijoint muscles and joints with stiffness. *Journal of Biomechanics*.

[30] Ma Y., Soatto S., Kosecka J., Sastry S. S. (2012). *An Invitation to 3-d Vision: From Images to Geometric Models*.

[31] Gareis H., Moshe S., Baratta R., Best R., D'Ambrosia R. (1992). The isometric length-force models of nine different skeletal muscles. *Journal of Biomechanics*.

[32] Kapandji A. (2007). *Physiologie articulaire-Schémas Commentés de Mécanique Humaine. Tome 3*.

[33] Brown S. H., McGill S. M. (2010). The relationship between trunk muscle activation and trunk stiffness: examining a non-constant stiffness gain. *Computer Methods in Biomechanics and Biomedical Engineering*.

[34] Dao T. T., Tho M. C. (2018). A systematic review of continuum modeling of skeletal muscles: current trends, limitations, and recommendations. *Applied Bionics and Biomechanics*.

[35] Maganaris C. N., Paul J. P. (1999). In vivo human tendon mechanical properties. *The Journal of Physiology*.

[36] Maganaris C. N., Paul J. P. (2002). Tensile properties of the in vivo human gastrocnemius tendon. *Journal of Biomechanics*.

[37] Magnusson S. P., Narici M. V., Maganaris C. N., Kjaer M. (2008). Human tendon behaviour and adaptation, in vivo. *The Journal of Physiology*.

[38] Zhibin S., Tianyu M., Chao N., Yijun N. (2018). A new skeleton model and the motion rhythm analysis for human shoulder complex oriented to rehabilitation robotics. *Applied Bionics and Biomechanics*.

[39] Chang M., O'Dwyer N., Adams R., Cobley S., Lee K. Y., Halaki M. (2020). Whole-body kinematics and coordination in a complex dance sequence: differences across skill levels. *Human Movement Science*.

[40] Rafique S., Najam-ul-Islam M., Shafique M., Mahmood A. (2020). Cartesian control of sit-to-stand motion using head position feedback. *Applied Bionics and Biomechanics*.

[41] Hlavenka T. M., Christner V. F., Gregory D. E. (2017). Neck posture during lifting and its effect on trunk muscle activation and lumbar spine posture. *Applied Ergonomics*.

